RETRACTED

# Correlations between chromobox homolog 8 and key factors of epithelial–mesenchymal transition in hepatocellular carcinoma

**DOI:** 10.1186/s12935-019-1063-z

**Published:** 2019-12-17

**Authors:** Xiaonian Zhu, Wei Luo, Chunhua Bei, Juan Kong, Shidong Zhang, Yuanyuan Fu, Di Li, Shengkui Tan

**Affiliations:** 1 Department of Epidemiology and Health Statistics, School of Public Health, Guilin Medical University, 109 Huancheng North Road 2, Guilin, 541004 Guangxi People’s Republic of China; 2 Nanchong Central Hospital, The Second Clinical College of North Sichuan Medical College, Nanchong, 637000 Sichuan People’s Republic of China

**Keywords:** Chromobox protein homolog 8, Hepatocellular carcinoma, Metastasis, Epithelial mesenchymal transition

## Abstract

**Background:**

Hepatocellular carcinoma (HCC) is one of the most common malignancies worldwide, especially in China, with high metastasis and poor prognosis. Recently, as the core component of the polycomb repressive complexes 1 (PRC1), chromobox protein homolog 8 (CBX8) is considered as an oncogene and prognostic marker in HCC.

**Methods:**

A tissue microarray of 166 paired HCC and adjacent non-tumor samples were collected to identify the relationship between CBX8 and epithelial mesenchymal transition (EMT) associated proteins by Spearman correlation analysis. Knock-down of CBX8 in HCC cells was conducted to detect the biologic functions of CBX8 in HCC metastasis.

**Results:**

We found out that CBX8 was over-expressed in HCC and its expression was closely related to the metastasis of HCC patients. In addition, knock-down of CBX8 was found to inhibit the invasion and migration ability of HCC cells. Moreover, there was a significant relationship between expression of CBX8 and EMT associated proteins both in HCC cells and tumor tissues.

**Conclusions:**

Our results indicate that CBX8 promotes metastasis of HCC by inducing EMT process.

## Background

Hepatocellular carcinoma (HCC) is one of the malignant tumors with the highest mortality rate. There are 841,000 new cases of HCC worldwide each year, and about 55% of HCC patients are from China [1]. Because of the high degree of malignancy and onset occult, most of HCC patients are diagnosed at late stage with poor outcome that the median survival time is only a few months [2, 3]. Though surgery and molecular targeted therapy of HCC develop fast and widely, high recurrence and high metastasis rate of HCC still results in very poor prognosis. Therefore, to find new predictive markers and identify their mechanism in metastasis become the key to improve the diagnosis and treatment of patients with HCC.

Polycomb group (PcG) proteins are essential regulators of cell proliferation and differentiation, which are often deregulated in human cancers and contribute to the development of cancers [4–6]. PcG proteins are primarily classified into two major protein complexes, named as the polycomb repressive complexes 1 and 2 (PRC1 and PRC2), whose function is to maintain transcriptional repression via chromatin remodeling and histone modification. In mammals, at least five different CBX proteins (CBX2, CBX4, CBX6, CBX7, and CBX8) are known to associate with the core PRC1 [7]. In our recent study, CBX7 has been found down-regulated in HCC tissues and related to HCC progression [8]. Moreover, we have also identified rs2289728 of *CBX4* and rs139394 of *CBX7* are protective single nucleotide polymorphisms (SNPs) to HCC [9].

RETRACTED

Chromobox homolog 8 (CBX8), a homologous to the Drosophila polycomb (Pc) protein, which is crucial for the pathogenesis of cancer indicated by recent reports. As a transcription repressor, CBX8 regulates numerous target genes important for cell growth and survival, including tumor suppressor gene INK4a/ARF locus [10] involved in cell-fate decisions and AF9 implicated in the development of acute leukemias [11]. CBX8 has been found up-regulated in human esophageal carcinoma, colorectal cancer and HCC [12–14]. Moreover, CBX8 is considered as an oncogene and prognostic marker in HCC [15].

As the most basic feature of tumor cells, invasion and metastasis are very important biological behavior of HCC. More and more evidence indicates that epithelial mesenchymal transition (EMT), an early sign of invasion and metastasis of tumors, is a vital process in tumor progression [16–18]. The main character of EMT is that cell morphology appears mesenchymal-like changes with the expression of cell adhesion molecules (such as E-cadherin and β-catenin) decreased and the expression of cytoskeleton vimentin proteins (such as Vimentin and N-cadherin) increased at the same time. Through EMT, epithelial cells lose cell polarity and weaken connection with basement membrane, resulting in malignant tumor cells to obtain higher ability of invasion and migration [19, 20]. So elucidating EMT process of tumor cells will be a great help to us to understand the metastasis of HCC clearly.

In this study, we find out that a significant relationship between the expression of CBX8 and EMT associated proteins in HCC cells and tumor tissues. Our results indicate that CBX8 plays a role in HCC metastasis by inducing EMT, suggesting CBX8 as a potential target in HCC treatment and prognosis.

## Materials and methods

### Antibodies and reagents

Antibodies against CBX8 (catalog No. ab182627), ZEB1 (catalog No. ab124512) and ZEB2 (catalog No. ab138222) were purchased from Abcam (Cambridge, MA, USA). Epithelial–mesenchymal transition (EMT) antibody sampler kit (catalog No. #9782) and phospho-β-catenin antibody (catalog No. #9561) were purchased from Cell Signaling Technology (Danvers, MA, USA). Anti-β-actin antibody (catalog No. 21800) was from Signalway Antibody LLC (College Park, Maryland, USA). Lipofecatmine 2000 (catalog No. 11668019) for cell transfection and Trizol (catalog No. 15596018) for RNA extraction were purchased from Thermo Fisher Scientific (Waltham, MA, USA). All other reagents were from Sigma-Aldrich (St. Louis, MO, USA) unless otherwise noted.

RETRACTED

### Patients and human tissue specimens

A total of 166 paired paraffin-embedded primary specimens from HCC patients under surgery during 2005 to 2009 were obtained from Department of Pathology, the Affiliated Hospital of Guilin Medical University. The patients were diagnosed according to their clinic-pathological characteristics. The clinic-pathological characteristics of these patients are shown in Additional file 1: Table S1. Another 31 pairs of fresh HCC tissues and the corresponding adjacent non-tumor tissues from the Affiliated Hospital of Guilin Medical University between 2014 and 2015 were stored at − 80 °C immediately after surgery and were used for semi-quantitative RT-PCR and Western blot. Informed consents were obtained from all patients and approved by the Institutional Research Ethics Committee of Guilin Medical University.

### Semi-quantitative RT-PCR

Total cell RNA was extracted by Trizol and reversed to cDNA for PCR using reverse transcription reagents (TIANGEN, Beijing, China). Then CBX8 and GAPDH were amplified by PCR and detected on a 1.5% agarose gel. PCR primers for CBX8 and GAPDH mRNA detection were as follows: CBX8 (F: 5′-TAAGGAAAGTAACACGGACCAA-3′, R: 5′-GAAATAAAAATCACTATGCCAA-3′), GAPDH (F: 5′-CCGCATCTTCTTTTGCGTCG-3′, R: 5′-AGTTAAAAGCAGCCCTGGTGA-3′).

### Western blot

Cells or powdered tissues were lysed in ice-cold RIPA buffer (Beyotime, Shanghai, China) containing protease inhibitors. After centrifugated at 12,000 rpm for 20 min at 4 °C, the lysates were resolved by SDS-PAGE and transferred to PVDF membranes. Then PVDF membranes were blocked in 5% fat-free milk in TBST for 1 h at room temperature. After washing with TBST for three times, primary antibodies with appropriate dilution were given and incubated at 4 °C overnight. The corresponding secondary antibodies were given the second day after TBST washing for three times. After incubated in secondary antibodies for 1.5 h at room temperature, the PVDF membranes were washed with TBST and detected by using ECL reagents (Beyotime).

### Immunohistochemical analysis and scoring

IHC staining for CBX8 and evaluation was performed in 166 paired paraffin-embedded HCC tissue specimens, and conducted by the same method as reported before [21].

RETRACTED

### Cell lines and shRNA transfection

Human hepatocytes (L02) and hepatic tumor cell lines (SK-Hep-1, HepG2, Hep3B, SMMC-7721, Huh-7, Bel-7402 and Li-7) were purchased from Cell Bank of Type Culture Collection of the Chinese Academy of Sciences (Shanghai, China), where they were characterized by DNA fingerprinting and isozyme detection. All the cell lines were revived every 3 to 4 months. SK-Hep-1, HepG2, Hep3B, SMMC-7721 and Huh-7 cells were cultured in Dulbecco’s modified Eagle medium (DMEM) with 10% fetal bovine serum (FBS). Bel-7402, Li-7 and L02 cells were cultured in RPMI-1640 medium with 10% FBS. All the cell lines were grown at 37 °C in a 5% CO_2_/95% air atmosphere.

Four lentiviral shRNAs targeting CBX8 (shCBX8) were synthesized on a GV248-puro vector (Genechem, Shanghai, China). Vector expressed GFP alone was used as a negative control (shGFP, provided by Genechem). According to the manufacturers’ instructions, CBX8 shRNAs were transfected into SK-Hep-1 cells using Lipofectamine 2000 reagent and detected after cultured for 2 to 3 days. Finally, shCBX8-1# (target sequence GGACGTGACCTCAAACTTT) and shCBX8-3# (target sequence TCGCTTGCTCGCAGCCTTT) were chosen for follow-up assays.

### Wound healing assay, cell invasion and migration analysis

The methods were also the same as reported before [21]. Briefly, Cells were seeded in 6-well plates and wounded by scratching with sterile plastic 10 μl micropipette tips. Cell migration distance was observed and photographed 0 h, 24 h and 48 h after the wounding by the phase contrast microscope. Cell invasion and cell migration were detected using Matrigel (BD, Franklin lakes, NJ, USA) coated or uncoated BD Transwell chamber, photographed and counted after crystal violet staining.

### Immunofluorescence

Cells were cultured in a 24-well plate for 24 h and then fixed with 4% formaldehyde. After that, cells were treated with 0.1% Triton X-100 and blocked in 5% FBS at room temperature. After incubated with primary antibodies overnight at 4 °C and secondary Goat Anti-Rabbit IgG H&L (Alexa Fluor^®^ 488, Abcam) antibodies for 1 h at 37 °C, cells were washed with PBS for 3 times and stained with DAPI for 5 min. Finally, the cells were observed and photographed under a fluorescence microscope.

### Statistical analysis

All statistical analyses were performed using SPSS version 19.0. The McNemar Chi square test was applied for the comparison of protein expression between HCC and corresponding adjacent non-tumor tissues. Correlations between CBX8 and EMT factors were analyzed by Spearman correlation test. The level of statistical significance was set at *P *< 0.05 for all tests.

RETRACTED

## Results

### CBX8 expression is associated with HCC metastasis

To confirm the role of CBX8 in metastasis for HCC patients, we first assessed CBX8 expression in a tissue microarray of 166 paired HCC and adjacent non-tumor samples. Immunohistochemical (IHC) assays showed that CBX8 was primarily localized in the nucleus. As shown in Fig. 1a, over-expression of CBX8 was found in HCC tissues, compared with adjacent non-tumor tissues. Especially, when we classified the HCC tissues according to distant metastasis, there was more CBX8 expression in metastatic HCC tissues than adjacent non-tumor tissues or non-metastatic HCC tissues. We further conducted semi-quantitative RT-PCR to detect the mRNA expression of CBX8 in 31 paired HCC and adjacent non-tumor tissues. As shown in Fig. 1b, the 9 cases of metastatic HCC tissues had a higher mRNA expression of CBX8 than adjacent non-tumor tissues or non-metastatic HCC tissues (*P *< 0.01). Up-regulation of CBX8 protein was confirmed in the same HCC samples by Western blot. Levels of CBX8 protein were significantly increased in HCC tissues, compared to the adjacent non-tumor tissues. And the metastatic HCC tissues had also a more expression of CBX8 protein than the non-metastatic HCC tissues (Fig. 1c, *P *< 0.01). Collectively, these results suggest that CBX8 is involved and functions in HCC metastasis.

**Fig. 1:** CBX8 is correlated with HCC metastasis. **a** Representative CBX8 protein expression was detected in adjacent non-tumor tissues, not metastatic and metastatic HCC tissues by immunohistochemical analysis at ×50 (upper panel) and ×400 magnification (lower panel). **b** Comparison of mRNA expression of CBX8 in adjacent non-tumor tissues, not metastatic and metastatic HCCs. **P < 0.01 is based on the Student *t* test compared to adjacent non-tumor tissues. **c** Comparison of protein expression of CBX8 in adjacent non-tumor tissues, not metastatic and metastatic HCCs. **P < 0.01 is based on the Student *t* test compared to adjacent non-tumor tissues

### Knock-down of CBX8 inhibits metastasis of HCC cells

In order to further clarify the biologic function of CBX8 in metastasis of HCC cells, we detected the expression of CBX8 protein in several HCC cell lines, SK-Hep-1, Bel-7402, Hep3B, Li-7, HepG2, Huh-7 and SMMC-7721. Compared with normal liver cell line L02, CBX8 was significantly increased in these HCC cell lines, especially in SK-Hep-1 and SMMC-7721 cells (Fig. 2a). At the same time, we purchased 4 shRNAs targeting CBX8 (shCBX8) and a negative control plasmid targeting GFP (shGFP). After introducing these shRNAs to SK-Hep-1 cell line, No.1# and 3# shCBX8 showed an ability of mRNA knock-down by more than 70% (Fig. 2b). Therefore, we selected SK-Hep-1 cell lines that had the relative high expression of CBX8 to construct CBX8 knock-down cells by introducing No.1# or 3# shCBX8 for the following study.

RETRACTED

**Fig. 2:** CBX8 promotes the metastasis of HCC cells. **a** CBX8 protein expression in L02 cell line and HCC cell lines as indicated was detected by Western blot (right panel, gray scan results normalized to β-actin). **b** CBX8 mRNA expression in SK-Hep-1 cells introduced with four specific shRNAs targeted CBX8 and a control shGFP by semi-quantitative RT-PCR (right panel, gray scan results normalized to GAPDH). **c** Invasion and migration ability of CBX8 knock-down cells was analyzed by wound healing. **P < 0.01 is based on the Student *t* test compared to shGFP cells. **d** Invasion and migration ability of CBX8 knock-down cells was analyzed by Transwell assay. **P < 0.01 is based on the Student *t* test compared to shGFP cells. All results are from three independent experiments

After that, we measured the invasion and migration ability of SK-Hep-1 cells after decreasing CBX8 expression. Wound healing assay was performed to detect tumor cell migration. As shown in Fig. 2c, wound area of SK-Hep-1-shCBX8 cells was significantly larger than control SK-Hep-1-shGFP cells at 48 h after wound time (*P *< 0.05). In accordance with the wound healing assay, both invasion and migration ability of SK-Hep-1 cells were significantly decreased when CBX8 expression was knocked-down in Transwell assay (*P *< 0.05, Fig. 2d). These results support that CBX8 promotes invasion and migration of HCC cells.

### CBX8 induces EMT process

Accumulated evidence indicates that EMT is a key process in HCC metastasis [22]. ERK and Wnt/β-catenin signaling pathways, E-cadherin, β-catenin, N-cadherin and Vimentin, are involved in EMT process and promote cancer metastasis [19, 23]. Therefore, we want to find out whether CBX8 can induce EMT to promote HCC cell invasion and migration by regulating EMT process. We purchased an EMT antibody kit to detect the expression of EMT associated factors in CBX8 knock-down cells. As shown in Fig. 3a, compared to the control SK-Hep-1-shGFP cells, epithelial markers β-catenin and E-cadherin were increased by 54% ± 10% and 161% ± 15%, while mesenchymal markers N-cadherin, Vimentin, zinc finger E-box binding homeobox 1 and 2 (ZEB1 and ZEB2), Snail and Slug were decreased by 75% ± 12%, 20% ± 9%, 68% ± 3%, 51% ± 15%, 65% ± 12% and 57% ± 19%, respectively in SK-Hep-1-shCBX8 cells. In addition, we found that phospho-β-catenin, an indicator of active β-catenin, was also increased after CBX8 knock-down, suggesting an increased nuclear localization of β-catenin in SK-Hep-1-shCBX8 cells. Furthermore, the Western blot result was also confirmed by immunofluorescence analysis that expression of EMT associated proteins changed by reducing CBX8 protein (Fig. 3b). These results show that CBX8 can regulate expression of EMT associated proteins.

RETRACTED

**Fig. 3:** CBX8 induces EMT. **a** Expression of EMT markers as indicated were detected in SK-Hep-1-shCBX8 cells by Western blot. **b** Expression of EMT markers as indicated were detected in SK-Hep-1-shCBX8 cells by immunofluorescence

### Correlations between CBX8 and EMT associated factors

Above findings led us to hypothesize that whether CBX8 exerts its function via EMT associated factors. Therefore, we detected the expression of EMT associated proteins in the 166 pairs of HCC and adjacent non-tumor tissues that CBX8 expression had been measured by IHC (Fig. 4a–f). In consistent with the early results, epithelial markers E-cadherin and β-catenin were decreased, while mesenchymal markers N-cadherin, Vimentin, ZEB1 and ZEB2 were significantly increased in HCC tissues, compared to the adjacent non-tumor tissues (*P *< 0.01, Table 1). In some HCC tissues, β-catenin transferred from cytoplasm to nucleus, which has been reported before [24]. In addition, in accordance with their roles in EMT process, we also found a significant correlation between ZEB1/ZEB2 and HCC metastasis [25]. We further analyzed the relationship between CBX8 and these EMT associated factors in the same 166 paired HCC tissues. As shown in Table 2, after Spearman correlation analysis, expression of CBX8 had a significant negative relationship with E-cadherin (r = − 0.446, *P *< 0.01) as well as β-catenin (r = − 0.530, *P *< 0.01), while a significant positive correlation with N-cadherin, Vimentin, ZEB1 and ZEB2 (r = 0.638, 0.473, 0.324, 0.402, all *P *< 0.01). The correlations between CBX8 and these EMT associated factors demonstrate that CBX8 induces EMT progression to promote metastasis of HCC.

**Fig. 4:** Expression of EMT associated factors in HCC tissues. **a–f** Representative expression of EMT markers as indicated was detected in HCC and adjacent non-tumor tissues by immunohistochemical analysis at ×50 (upper panel) and ×400 magnification (lower panel)

**Table 1:** Expression of EMT factors in paired HCC and adjacent non-tumor tissues

HCC tissues	n	Adjacent non-tumor tissues		*P* value
		High	Low	
E-cadherin				
High	54	23	31	*0.008*
Low	112	72	40	
β-catenin				
High	69	50	19	*0.001*
Low	97	46	51	
N-cadherin				
High	79	33	46	*0.005*
Low	87	22	65	
Vimentin				
High	117	56	61	*0.000*
Low	49	15	34	
ZEB1				
High	121	67	54	*0.000*
Low	45	17	28	
ZEB2				
High	102	48	54	*0.000*
Low	65	20	45	

Italic values indicate significance. *P* value is based on the McNemar χ^2^ test

RETRACTED

**Table 2:** The correlation between CBX8 and EMT factors in HCC tissues

EMT factors	n	CBX8		χ^2^ value	r value	*P* value
		High	Low			
E-cadherin						
High	54	9	45	33.066	− 0.446	*0.000*
Low	112	72	40			
β-catenin						
High	69	12	57	46.608	− 0.530	*0.000*
Low	97	69	28			
N-cadherin						
High	79	65	14	67.637	0.638	*0.005*
Low	87	16	71			
Vimentin						
High	117	75	42	37.172	0.473	*0.000*
Low	49	6	43			
ZEB1						
High	121	71	50	17.447	0.324	*0.000*
Low	45	10	35			
ZEB2						
High	102	66	36	26.805	0.402	*0.000*
Low	64	15	49			

Italic values indicate significance. *P* value is based on Spearman correlation test

## Discussion

HCC is one of the most common malignant tumors with high mortality rate worldwide [26], because of its insidious onset, frequent metastasis and high recurrence rate after surgery. Various genetic and epigenetic changes have been identified in the occurrence and progression of HCC, such as *p53*, β-catenin and TGF-β [27, 28]. Both *p53* deficiency and mutation contribute to HBV- and HCV-related HCCs [29]. As a crucial downstream component of the Wnt signaling pathway, mutations and increased nuclear expression of β-catenin have been detected in human HCC specimens [30]. And TGF-β modulates various microenvironment factors involved in HCC through intrinsic or extrinsic signaling pathway [31]. In this study, we clarify a significant correlation between expression of CBX8 and EMT associated markers in HCC cells and tissues, supporting a role of CBX8 playing in HCC progression and metastasis.

CBX8 is the core component of the PRC1 complex and directly regulates expression of various target genes. CBX8 was early discovered to be involved in regulation of cell senescence through binding to INK4a/ARF locus [10]. In addition, CBX8 was found to be induced by oxidative damage of DNA, and the damage got worse when CBX8 was silenced, indicating CBX8 was a DNA repair protein [13, 32]. Moreover, recent studies have shown that CBX8 was deregulated in several kinds of tumors including HCC. CBX8 was over-expressed in HCC tissues and correlated with poor prognosis of patients [14, 15]. Mechanistically, CBX8 activates bone morphogenetic protein 4 (BMP4) transcription by modulating H3K27me3 [15]. In addition, CBX8 could efficiently activate AKT/β-catenin signaling via up-regulation of the transcription factor EGR1 and miR-365-3p [14].

Invasion and metastasis is an important biological feature of malignant tumors. Various molecules and pathways are involved in the process of tumor metastasis and invasion. EMT is a biological process that epithelial cells acquire mesenchymal phenotype by specific steps and plays a key role in tumor invasion and metastasis [33]. EMT promotes cancer cells to be more aggressive and causes a series of consequences, such as drug resistance, apoptotic inhibition and immunologic deficiency [34]. Furthermore, the EMT in cancer cells is a dynamical process and transits between the epithelial, partial-EMT and mesenchymal states. Partial-EMT, a state of epithelial and mesenchymal markers concurrently express in cancer cells, was recently recognized to pose a higher metastatic risk rather than complete EMT [35]. To clarify the mechanism of tumor cell proliferation and the induction of EMT will provide a great help to understand the metastasis of HCC. We measured expression of EMT markers in HCC cells and tissues, including E-cadherin, β-catenin, N-cadherin, Vimentin, ZEB1 and ZEB2. Accumulated evidence shows that ZEB1 and ZEB2 are involved in EMT process as two key mesenchymal markers. ZEB1 and ZEB2 were both reported to inhibit expression of E-cadherin [36], and induce EMT process to promote tumor invasion and migration [37]. Finally, we confirmed that CBX8 promoted HCC metastasis by regulating expression of EMT markers. In accordance with other reports [24, 38–40], we found these EMT markers were deregulated in HCC tissues. Furthermore, we identified a significant correlation between CBX8 and these EMT markers.

RETRACTED

## Conclusions

In a conclusion, we clarify that CBX8 induces EMT process in HCC, which is in consistent with the correlation between its high expression and EMT associated markers. Our results indicate that CBX8 is likely to become a new therapeutic target of HCC.

## Supplementary information

**Additional file 1: Table S1.** Correlation between CBX8 expression and clinic-pathological characteristics of HCC patients.

## Data Availability

All data generated or analysed during this study are included in this published article and its additional files.
